# The Efficacy and Safety of Budesonide/Glycopyrronium/Formoterol in the Treatment of COPD in the Elderly

This article has been retracted.

**DOI:** 10.1155/2022/8382295

**Published:** 2022-08-17

**Authors:** Min Guo, Chuan Yu, Zenian Li

**Affiliations:** Department of Respiration, General Hospital of Pingxiang Mining Industry Group Co., Ltd, Pingxiang 337000, China

## Abstract

**Objective:**

Chronic obstructive pulmonary disease (COPD) is a major and difficult disease of the chronic respiratory system that is common and frequent, with a huge disease burden. The aim of this study was to investigate the efficacy and safety of budesonide/glyburide/formoterol fumarate (BGF) in the treatment of COPD.

**Methods:**

A comprehensive literature search was conducted in PubMed, Embase, Cochrane Library, and Web of Science. The basic features of the seven pieces of literature were identified using the search strategy. The sample size range was 130∼1264.

**Results:**

The effects of BGF increased FEV1 in patients with COPD (mean difference = 2.86, 95%CI: 2.71–3.01, *p* < 0.00001). The effects of BGF improved in patients with ≥1 TEAE in patients with COPD, and was not statistically significant after treatment (Odds rate = 1.00, 95%CI: 0.85–1.17, *p*=0.97). The effects of BGF increased in patients with TEAEs related a to study treatment in patients with COPD (odds rate = 1.27, 95% CI: 1.03–1.57, *p*=0.02). The effects of BGF in decreased patients with serious TEAEs in patients with COPD (odds rate = −0.02, 95% CI: −0.03–−0.00, *p*=0.04). The effects of BGF decreased the death rate in patients with COPD, and were not statistically significant after treatment (odds rate = 0.77, 95% CI: 0.31–1.97, *p*=0.59). The effects of BGF decreased the hypertension rate in patients with COPD (odds rate = 0.92, 95% CI: 0.44–1.89, *p*=0.81), and was not statistically significant after treatment. The effects of BGF increased pneumonia in patients with COPD (odds rate = 1.55, 95% CI: 0.81–2.97, *p*=0.19), and were not statistically significant after treatment. The effects of BGF increased FEV1, increased patients with TEAEs related a to study treatment, and decreased patients with serious TEAEs in patients with COPD.

**Conclusion:**

This study elucidates the efficacy and safety of BGF in the treatment of COPD with a view to providing a clinical reference.

## 1. Introduction

Chronic obstructive pulmonary disease (COPD) is a common, frequently occurring, major, and difficult disease of the chronic respiratory system [1]. It has a huge disease burden and has attracted more and more attention in recent years [2]. The number of COPD patients in the world is about 3 8.4 billion, ranking the fourth cause of death in the world [3]. The WHO estimates that it will rise to the third place in 2020. 3 million people die of COPD every year in the world [4]. It is estimated that 4.5 million people will die from COPD related diseases every year in 2030 [4]. Chronic obstructive pulmonary disease is becoming more and more serious worldwide [5]. COPD ranks third as the leading cause of death in China, with a total number of patients of about 100 million people [6]. According to the global disease burden data, in 2016, the number of COPD deaths in China (876300) accounted for 29.5% of the total number of COPD deaths in the world 86% [7]. According to the 2019 study of mortality, incidence rate, and risk factors in China and its provinces, the Lancet published in 2019 showed that chronic obstructive pulmonary disease (LPG) has become the top five health burden among Chinese residents, ranking third as the largest cause of death and loss of life in China [8]. The prevention and treatment measures of COPD include prevention, early diagnosis, and standardized treatment (drug treatment, exercise therapy, psychological intervention, lung rehabilitation, etc.), and lung rehabilitation is an integral part of it [7, 8].

With the development of the social economy, air pollution has become a serious public health problem all over the world, which seriously endangers the health of residents and leads to a heavy burden of disease [9]. Atmospheric particulate matter is an important part of air pollutants. In recent years, its relationship with an acute attack and death of respiratory diseases has been explained [9].

COPD is a disease that can be prevented and treated with the characteristics of airflow restriction [10]. Airflow restriction is not completely reversible and develops continuously, which is related to the abnormal inflammatory response of the lungs to harmful gases or particles such as cigarettes and smoke [11]. Due to the large number of patients, high mortality, and heavy social and economic burden, the disease has become an important public health problem [12]. According to statistics, COPD will become the fifth disease to cause an economic burden in the world by 2020 [13]. In recent years, a large number of scientific studies have deeply analyzed and explored its pathogenesis, and remarkable progress has been made [12].

Budesonide is a steroid hormone which can increase the level of endogenous corticosteroids and has a significant anti-inflammatory activity [14]. It is a hormone that can be inhaled by aerosol [14]. Budesonide is a glucocorticoid with high-efficiency and a local anti-inflammatory effect [15]. It can enhance the stability of endothelial cells, smooth muscle cells, and lysosomal membrane, inhibit immune response and reduce antibody synthesis, so as to reduce the release and activity of allergic active mediators such as histamine, reduce the enzymatic process stimulated by antigen antibody binding, inhibit the synthesis and release of bronchoconstrictor substances and reduce the contraction reaction of the smooth muscle [16]. Clinically, it is used in patients with glucocorticoid-dependent or independent bronchial asthma and asthmatic chronic bronchitis [17]. Glycopyrronium bromide is a long-acting quaternary ammonium muscarinic receptor antagonist [18]. Its selectivity to the human M3 receptor is more than 4 times that to the human M2 receptor [19]. The most common adverse reaction of glycopyrronium bromide was dry mouth, but most of them were mild rather than severe; other common adverse reactions include gastrointestinal reactions (including gastroenteritis and dyspepsia), local adverse reactions (laryngitis, rhinitis, rhinitis, and sinusitis), eye problems (pupil dilation and blurred vision), palpitation and arrhythmia (atrial fibrillation^*∗*^), urinary symptoms (urinary tract infection, dysuria, and urinary retention), and limb pain, chest pain, caries, rash, headache, insomnia, and cognitive impairment [19–21].

Formoterol fumarate is a bronchodilator, which can effectively relax the airway smooth muscle, relieve airway obstruction, and quickly improve symptoms such as dyspnea [22]. Relevant studies have pointed out that the combination of formoterol fumarate and tiotropium bromide can further enhance the therapeutic effect of COPD and accelerate the improvement of pulmonary function [23–25]. This study was aimed to explore the efficacy and safety of budesonide/glycopyrronium/formoterol fumarate in the treatment of COPD.

## 2. Materials and Methods

### 2.1. Literature Search

The experiment was searched from PubMed, Embase, and Web of Science, and the last search was performed on March 2022. The free words adopted were as follows: “budesonide/glycopyrronium/formoterol fumarate,” “chronic obstructive pulmonary disease,” “budesonide,” “glycopyrronium,” “formoterol fumarate,” and their combinations. The reference lists of previous relevant reviews were manually checked to find additional publications of interest. The language of publications was restrained to English.

### 2.2. Inclusion and Exclusion Criteria

The following inclusion criteria were used to select eligible studies: (i) the diagnosis of cerebral infarction was pathologically confirmed; (ii) the forced expiratory volume in one second (FEV1) and safety population (death rate, hypertension rate, or pneumonia) were evaluated in this study. The exclusion criteria were as follows: (i) abstract, review, case report, or comment letter; (ii) animal studies; (iii) duplicate publications; (iv) published not in English or Chinese.

### 2.3. Data Extraction

Two independent reviewers using a standardized form extracted relevant data from eligible studies as literature [26]. Data were analyzed by using Review Manager 5.3 as literature [26]. Heterogeneity among studies was examined using the chi-square-based *Q* test in which I2 indicates the level of heterogeneity. I2 < 50% or pheterogeneity>0.1 represented low heterogeneity. *p* < 0.05 was considered statistically significant.

## 3. Results

### 3.1. Features of Included Studies

This study was identified through systematic literature searching. 531 pieces of literature were identified and evaluated. The literature selection process is shown in Figure 1. The basic features of 7 studies [27–33] are shown in Table 1. The sample size ranged from 130 to 1264.

### 3.2. Characteristics of the Included Studies

The quality of literature was evaluated using the Cochrane Collaboration's tool for assessing risk of bias (Figures 2(a) and 2(b)). The numerous numbers of studies were randomized, properly allocated with concealment strategies, and reported incomplete outcome data and double-blind (Figures 2(a) and 2(b)), as shown in Figure 2.

### 3.3. The Effects of BGF on FEV1 of COPD

The study analyzed the effects of BGF on FEV1 of COPD. As shown in Figure 3(a), the effects of BGF increased FEV1 in patients with COPD (mean difference = 2.86, 95%CI: 2.71–3.01, *p* < 0.00001), as shown in Figure 3.

### 3.4. The Effects of BGF on TEAEs of COPD

The study analyzed the effects of BGF on TEAEs of COPD. As shown in Figure 4(a), the effects of BGF increased in patients with ≥1 TEAE in patients with COPD, and were not statistically significant after treatment (odds rate = 1.00, 95%CI: 0.85–1.17, *p*=0.97). As shown in Figure 4(b), the effects of BGF increased in patients with TEAEs related a to study treatment in patients with COPD (odds rate = 1.27, 95%CI: 1.03–1.57, *p*=0.02). The effects of BGF decreased in patients with serious TEAEs in patients with COPD (Odds rate = −0.02, 95%CI: −0.03–−0.00, *p*=0.04, Figure 4(c)), as shown in Figure 4.

### 3.5. Publication Bias for FEV1 or TEAEs of COPD

Funnel plots for meta-analysis of FEV1 or TEAEs of cerebral infarction are shown in Figures 3(b) and 5. The funnel plots for all analysis were symmetric, indicating no obvious publication bias, as shown in Figure 5.

### 3.6. The Effects of BGF on Safety Population of COPD

The study analyzed the effects of BGF on the safety population of COPD. As shown in Figure 6(a), the effects of BGF decreased the death rate in patients with COPD, and were not statistically significant after treatment (odds rate = 0.77, 95%CI: 0.31–1.97, *p*=0.59). As shown in Figure 6(b), the effects of BGF decreased the hypertension rate in patients with COPD (odds rate = 0.92, 95%CI: 0.44–1.89, *p*=0.81), and were not statistically significant after treatment. The effects of BGF increased pneumonia in patients with COPD (odds rate = 1.55, 95%CI: 0.81–2.97, *p*=0.19, Figure 6(c)), not statistically significant after treatment, as shown in Figure 6.

### 3.7. Publication Bias for Safety Population of COPD

Funnel plots for meta-analysis of FEV1 or safety population of cerebral infarction are shown in Figure 6. The funnel plots for all analysis were symmetric, indicating no obvious publication bias, as shown in Figure 7.

## 4. Discussion

Chronic obstructive pulmonary disease (COPD) has been widely concerned by medical circles all over the world because of its high prevalence, high mortality, and high disability rate [34]. At present, reducing the probability of premature death caused by chronic respiratory diseases represented by chronic obstructive pulmonary disease has been identified as one of the important indicators of “Healthy China 2030” [35]. Our results showed that 7 pieces of literature published from 2017 to 2021 with 2718 patients were included in meta-analysis.

Population aging is one of the main problems China is facing at present [36]. It is estimated that by 2050, China's population over the age of 60 will reach 498 million [37]. The incidence rate of pulmonary fibrosis and chronic obstructive pulmonary disease is also increasing gradually with the increase of age [38]. The occurrence and development of these diseases are closely related to aging. Some changes in the structure and molecular phenotype of aging may participate in this process [39]. In addition, at present, the treatment of pulmonary fibrosis and chronic obstructive pulmonary disease mainly includes nondrug management (pulmonary rehabilitation, oxygen supplement, and surgical treatment) and drug management (glucocorticoids, immunosuppressants, bronchodilators, and targeted drugs) [38]. However, these treatment methods also have many disadvantages [40]. For example, in nondrug management, patients are rarely able to carry out lung rehabilitation training as required, and the source and rejection of lung transplantation are great problems; in drug management, the application of glucocorticoids and immunosuppressants will lead to many complications and cannot reverse the existing lesions [41, 42]. The use of bronchodilators has not been proved to effectively prolong the survival of patients and has the limitations of targeted drugs [43]. These results of meta-analysis showed that the effects of BGF increased FEV1 in patients with COPD (mean difference = 2.86, 95%CI: 2.71–3.01, *p* < 0.00001).

The development of chronic obstructive pulmonary disease is a complex, multielement, and multiring process [44]. Chronic airway inflammation, protease/antiprotease imbalance, oxide/antioxidant imbalance, autoimmunity, apoptosis, and gene polymorphism are all involved in the occurrence and development of chronic obstructive pulmonary disease. It can provide an important basis for finding better treatment and early prevention measures in clinics [45, 46]. These results of meta-analysis showed that the effects of BGF increased in patients with TEAEs related a to study treatment in patients with COPD (odds rate = 1.27, 95%CI: 1.03–1.57, *p*=0.02). The effects of BGF decreased in patients with serious TEAEs in patients with COPD (odds rate = −0.02, 95%CI: −0.03– −0.00, *p*=0.04).

With the growth of age, the incidence of many lung diseases is also gradually increasing, among which chronic obstructive pulmonary disease and pulmonary fibrosis are the most significant [47]. At present, some progress has been made in the relationship between aging, and chronic obstructive pulmonary disease and pulmonary fibrosis [48]. However, the specific molecular mechanism and functional relationship of aging in the occurrence and the development of chronic obstructive pulmonary disease and pulmonary fibrosis are not completely clear [49]. Finding these molecular mechanisms and functional relationships may bring hope to cure these diseases [50]. The present study showed that the effects of BGF did not have significant effects on the death rate, hypertension rate, and pneumonia in patients with COPD.

The present study has some limitations. First, all citations only researched that the effects of BGF increased FEV1 in patients with COPD. Second, due to a relatively low number of studies included depicted the relationship between BGF and the treatment of COPD, which is an important reason for the heterogeneity of this results. It is necessary to develop high-quality large-scale studies with more complete patients' types to verify our results. Finally, significant heterogeneity was detected for several parameters, however, we used the fixed-effect model according to heterogeneity, which also existed due to the difference in included studies.

## Figures and Tables

**Figure 1:** Features of included studies.

**Figure 2:** Characteristics of included studies. Risk of bias summary (a). Risk of bias graph (b).

**Figure 3:** The effects of BGF on FEV1 of COPD. Forest plot (a), and publication bias for FEV1 (b).

**Figure 4:** The effects of BGF on TEAEs of COPD. A forest plot for patients with ≥1 TEAE (a), patients with TEAEs related a to study treatment (b), and patients with serious TEAEs (c).

**Figure 5:** Publication bias for TEAEs of COPD. Publication bias for patients with ≥1 TEAE (a), patients with TEAEs related a to study treatment (b), and patients with serious TEAEs (c).

**Figure 6:** The effects of BGF on the safety population of COPD. Forest plot for death rate (a), hypertension rate (b), and pneumonia (c).

**Figure 7:** Publication bias for safety population of COPD. Publication bias for death rate (a), hypertension rate (b), and pneumonia (c).

**Table 1:** Basic characteristics of included studies.

Study year	Country	Ethnicity	Cases	Gender (M/F)
Darken 2018	USA	America	160	81/79
Ichinose 2019	Sweden	Europe	277	139/138
Ichinose-2 2019	Sweden	Europe	1277	139/138
Maes 2017	USA	America	130	64/66
Martinez-1 2021	USA	America	322	170/152
Muro 2021	Japan	East Asia	1264	639/625
Wang 2020	China	East Asia	288	144/144

## Data Availability

The simulation experiment data used to support the findings of this study are available from the corresponding author upon request.
